RETRACTED

# A Study on Parents' Attitudes towards Middle School Students' Online Learning Based on Statistical Analysis

**DOI:** 10.1155/2022/4848738

**Published:** 2022-06-21

**Authors:** Guomin Chen, Shihui Zheng, Jianwu He, Xiaowei Wang

**Affiliations:** ^1^Guilin University of Aerospace Technology, Guilin, China; ^2^School of Economics and Management, Dalian University of Techonology, Dut School of Economics and Management, Dalian, China; ^3^College of Tourism and Landscape Architecture, GUT, Guilin, China; ^4^Dalian University of Finance and Economics, Dalian, China

## Abstract

Based on the role separation scenario in which students need parental support, this paper explores the effect of parents' attitude on secondary school students' online learning. Through structural equation model analysis and regression analysis of 745 valid responses to a questionnaire, the data results show that parents' subjective dimension includes perceived gain and perceived loss, and social factor dimension includes teachers' influence and online comments. Perceived value is the key influencing factor of parents' attitude towards secondary school students in online learning platform. Perceived usefulness and platform information influence parents' attitude positively and significantly, while perceived risk influences parents' attitude negatively and significantly. In the dimension of social factors, teachers' influence positively influences parents' attitude, and online comments modulate the influence of perceived value on parents' attitude.

## 1. Introduction

Since COVID-19 broke out globally in 2020 and is expected to coexist with humans for some time to come, countries have started online learning. Online learning has gradually changed from the role of auxiliary teaching to the leading role of stage teaching and has received unprecedented attention and rapid development, so online learning has become the new normal in the learning of middle school students.

The research is focused on parents' attitudes towards students' use of online learning platforms. Most middle school students in China are teenagers aged between 12 and 18 with a certain subjective awareness of learning. As direct users of online learning platforms, they have their own feelings about the platform, and their choice of online learning platforms is more influenced by parents' attitudes. This leads to the separation of direct users (middle school students) and indirect users (parents). Although there are extensive researches on online learning platforms at present, the research on parents' attitudes towards students' use of online learning is still in the blank stage, which makes this research of great significance.

RETRACTED

## 2. Variables and Research Hypothesis

### 2.1. Perceived Usefulness and Perceived Value: Parent Attitude

In information systems and technology research, perceived usefulness has been broadly used as a key indicator for predicting technology reception. Keng-boon Ooi et al. reported that perceived usefulness, perceived ease of use, and belonging have an obvious direct effect on satisfaction, while satisfaction directly affected learners' website attachment and continuous use [1]. Chang et al. investigated the influencing factors of behavioral intention of e-learning for educational purposes among Azerbaijani college students, finding a strong beneficial impact of perceived usefulness on college students' attitude toward using e-learning [2]. Zhang who conducted a study on user selection factors of online Chinese education in Thailand found that perceived usefulness does not leave any direct impact on respondents' willingness of the online learning Chinese in Russia but indirectly affects the perceived value, which is one of the highest path coefficients, suggesting the mediating effect of perceived value on perceived usefulness on adoption intention [3]. For online learning, perceived usefulness is an important direct factor influencing customer attitudes, or indirectly through perceived value. The effect of perceived usefulness on perceived value and parents' views is investigated in this paper using perceived usefulness as an antecedent variable for perceived value. This paper proposes the following hypotheses:

  H1: Parents' perceived usefulness of e-learning platforms positively affects parents' attitudes.
  H2: Parents' perceived usefulness of e-learning platforms positively affects parents' perceived value.

### 2.2. Platform Information and Perceived Value: Attitudes of Middle School Students' Parents

For users, information serves as a provider as well as a recommender. Information can serve as a provider of relevant product or service material to users, as well as a recommender to assist them in making decisions [4]. Customers can make better selections when purchasing online if they have access to a number of objective product information [5]. Yang et al. found that the online and offline information integration significantly promotes perceived profit. Correspondingly, perceived profit positively affects perceived value and indirectly influences usage attitudes through it when conducting the influence of physical experience and information integration on consumers' use of conventional commerce and e-commerce [6]. The platform information for students and parents provides an important basis for shaping consumers' perceived value and attitude while building an online learning platform. The platform information can not only provide students and parents with the information they need about the platform services and courses, but also assist parents to make decisions on whether to let students continue to use the online learning platform. The following hypotheses are thus proposed:

  H3: The information of online learning platform positively affects the attitudes of parents of middle school students.
  H4: The information of online learning positively affects the perceived value of parents of middle school students.

RETRACTED

### 2.3. Perceived Risk and Perceived Value: Parents' Attitudes of Middle School Students

Uncertainty, loss, and lack of control for a product or service are all examples of perceived risk. Foreign studies have verified the repeated negative effect of perceived risk on mobile services' perceived value [7], mobile payment's perceived value [8], utilitarianism, and hedonic value in B2C e-commerce. Domestic studies have also reached similar conclusions. When Yan looked at the elements that influence college students' desire to accept MOOCs, she discovered that perceived risk, as portion of perceived profit and loss, has a negative and significant effect on perceived value [9]. Jiang found that perceived risk negatively significantly affects perceived value and trust when conducting research on factors influencing mobile O_2_O application attitude [10]. There is a general consensus at home and abroad that perceived risk can have a marked negative effect on perceived value. Customers, on the other hand, tend to avoid risks in unclear situations, and parents of middle school students who use online learning platforms similarly tend to avoid risks when taking decision. Perceived risk causes a detrimental effect to product/service perceived value and attitude in general. This paper proposes the following hypotheses:

  H5: Perceived risk negatively affects parents' perceived value for online learning platforms.
  H6: Perceived risk negatively affects the attitudes of parents of middle school students for online learning platforms.

### 2.4. Perceived Cost and Perceived Value: Attitudes of Middle School Students' Parents

Perceived cost (also known as perceived price) is a key component influencing customer demand, user acceptance, and innovation implementation in many information systems, marketing, and economic models. Perceived cost generates an adverse effect on perceived value at the judgment stage under the monetary standpoint. Wang et al. examined the adoption of mobile hotel booking (MHR) from the value and found that perceived value was the predictor of customer adoption of MHR. In terms of perceived profit and loss, technical effort and perceived cost significantly affect perceived value [11]. Wang et al. investigated the determinants of mobile app users' behavioral intention based on the consumption value theory, and the results showed that consumption value greatly influenced the behavioral intention of consumers in using mobile applications. Among them, affective value and cognitive value have strong relationship with behavioral intention. Furthermore, by the mediating effect of other consumption values (functional value, social value, emotional value, and cognitive value), conditional value affects mobile app users' behavioral intention [12]. This paper proposes the following hypotheses:

  H7: Perceived cost negatively affects parents' perceived value for online learning platforms.
  H8: Perceived cost negatively affects parents' attitudes towards online learning platforms.

RETRACTED

### 2.5. Teachers' Influence and Perceived Value: Parents' Attitudes of Middle School Students

New users have less product or service knowledge and no prior experience than existing users. As a result, new users are more likely to base their decisions on the evaluation and social recognition of reference groups. The research by Huang explores how social features and interaction affect users' online experience, supporting the usage of stimulus-organic-response (S-O-R) models in social network sites. The study also demonstrates ways to integrate environmental features to enhance the online experience and purchase intention of users [13]. Cheung et al.'s study explores how members of virtual Internet platforms assess their knowledge sharing experiences and how such assessments affect their decision of continually sharing knowledge in online practice communities. It turns out that members are satisfied when they receive the reciprocity that they anticipate. Similarly, they will be delighted, and their knowledge self-efficacy can be strengthened if they discover that they can support other members according to their expectations [14]. Parents of middle school students seem to be more cautious in selecting and using digital training platforms for their children when they pay greater attention to their students' education. Teachers are the most important reference group, and parents will pay more attention to teachers' recognition and suggestions on online learning platforms. This paper suggests the following hypotheses based on existing research findings:

  H9: The perceived value of online learning platforms from parents of middle school students was positively affected by teacher influence.
  H10: The attitudes towards online learning platform from parents of middle school students were positively affected by teacher influence.

RETRACTED

### 2.6. Online Comments and Perceived Value: Parents' Attitudes of Middle School Students

In this information-rich society, customers' decisions are often made in the context of the whole social environment. Online comments on products or services (which tend to be online information exchange between strangers) should be considered [15]. The perceived risks and uncertainties can be efficiently minimized through referring to online reviews [16]. Consumers believe that online reviews, whether positive or negative, offered by product or service suppliers are preferable to information provided by online reviews. These will be used as a key reference point in decision-making [17]. Studies have shown that customer behavior is influenced by online comments [18–20]. Customers can use online comment information as a source of real reference information to affect their decision-making behavior. As online learning platforms continually grow, the companies try to seek means to utilize online reviews to affect client attitudes, as well as altering their marketing tactics based on the results of online reviews. This paper proposes the following hypothesis:

  H11: Online comments positively moderate perceived value and parents' attitudes on online learning platforms.

### 2.7. Perceived Value and Parents' Attitudes of Middle School Students

According to the empirical study with 222 young adult SMS users, Turel et al. found that perceived value was a critical multidimensional determinant for behavioral intention [21]. Yang and Jolly investigated how consumers' perceived value and subjective norms affected their use of mobile data services in the United States and South Korea. The negative impacts of the four categories of customer perceived value were discovered to reflect distinct behavioral intents to utilize mobile data services in these two nations. Emotional value has the greatest impact on consumer use of mobile data services in both nations. Subjective norms are an important anther factor of American consumers' attitude and behavioral intention for the use of mobile data services, while they are insignificant among Korean consumers [22]. Hong et al.'s study analyzed the influencing factors of persistence attitude of smart watches and found that persistence intention is directly influenced by hedonic value and utilitarian value of perceived value [23]. According to research, the perceived value of Internet items or services has a positive effect on behavioral intentions to use and acquire them. In essence, middle school students' learning behavior on online learning platforms is to gain an educational environment and learning services and relevant information from associated online products. This paper proposes the following hypothesis:

  H12: Perceived value positively affects the attitudes of parents of middle school students towards online learning platforms.

RETRACTED

To sum up, the authors put forward the research hypothesis of this paper after reasoning analysis, as shown in Table 1.

## 3. Research Model and Design

### 3.1. Research Model

Through sorting out the relation of variables included in the current studies, the attitude model for middle school students' parents under the perceived value theory is finally determined and formed. Perceived value theory is generally thought to be made up of two parts, perceived gains and perceived benefit, so the independent variables of perceived usefulness, platform information, perceived risk, and perceived cost are classified as variables affecting perceived gain in perceived value (perceived usefulness and platform information) and the variables that affect perceived loss (perceived risk and perceived cost). External situational variables include teachers' influence and adjustment of the variables in the independent variable network comments. Teachers' influence is closely related to the user of the key groups opinion on its attitude, while network review focuses on the new groups for the comments and opinions of products required for the influence of parents' attitude, combined with the perceived value model (VAM), to generate the theoretical model for the current research.  Figure 1 exhibits the hypothesis relation and model.

### 3.2. Measurement Scales

For ensuring measurement scale reliability and validity, the variables to be measured are all used in the existing mature measurement scale in the existing literature, and appropriate adjustments are made according to the research purpose and research situation of this paper, so as to be used as a measurement tool for data collection. All questions related to the structure of the paper used a 5-point Likert scale, in which 1 represented “disagree” and 5 represented “agree.” Based on the relationship between variables studied, this paper divides them into independent variables, mediating variables, moderating variables, and dependent variables. The specific dimensions and measurement items are as follows.

#### 3.2.1. Measurement of Independent Variables

① Perceived usefulness
  In the context of the current research, perceived usefulness means the extent to which parents of secondary school students perceive that the content of the curriculum matches the needs of their children. For measurement, a 5-point Likert scale was used, in which (1) represented “strongly disagree” and (5) represented “strongly agree.” Perceived usefulness is the independent variable of perceived gains, and the three questions are adapted from the scale of Davis [24], as seen in Table 2.
② Platform information
  In the current research, platform information refers to the detailed introduction of learning resources, course arrangement, teaching content, and other relevant information on the network by the online learning platform in order to attract users, enhance user experience and shape, and maintain high-quality user relationship. For measurement, a 5-point Likert scale was used, in which (1) represented “strongly disagree” and (5) represented “strongly agree.” Platform information is the independent variable of perceived gain, and the three questions are adapted from the scale of Li [25], as shown in Table 3.
③ Perceived risk
  The perceived risk in this study refers to customers' awareness of the significance of the potential downside consequences of using the incorrect e-learning product and the probability of making the poor decision in an e-commerce setting. For measurement, a 5-point Likert scale was used, in which (1) represented “strongly disagree” and (5) represented “strongly agree.” Perceived risk is the independent variable of perceived profit and loss, and the three items are adapted from Zhao et al. [26], as shown in Table 4.
④ Perceived cost
  In this study, perceived cost refers to the cost perceived by middle school students to purchase learning equipment, pay Internet fees, or go to Internet cafes for learning on the online learning platform. A 5-point Likert scale is adopted for measurement, in which (1) represented “strongly disagree” and (5) represented “strongly agree.” Perceived cost is the independent variable of perceived profit and loss, and the four questions are adapted from Wang et al. [27], as shown in Table 5.
⑤ Teacher influence
  In this study, teacher influence refers to the influence of teachers in students' real schools on parents' attitudes towards students using online learning platforms. A 5-point Likert scale is adopted for measurement, in which (1) represented “strongly disagree” and (5) represented “strongly agree.” The four questions of teacher influence are adapted from Ashwin et al. [28], as shown in Table 6.

RETRACTED

#### 3.2.2. Measurement of Dependent Variables

As the dependent variable of this study, parent attitude refers to the stable psychological tendency of middle school students' parents towards the use of online learning platforms. In the design process of this study, parent attitudes towards online learning platforms are mainly influenced by independent variables directly and indirectly through perceived value. A 5-point Likert scale is adopted for measurement, in which (1) represented “strongly disagree” and (5) represented “strongly agree.” Three items for parent attitudes are based on the version of Raghu et al. [29] and appropriately adjusted according to the context that is easy for parents to understand on the online learning platform, as shown in Table 7.

#### 3.2.3. Measurement of Intermediary Variables

Perceived value is the mediating variable of this study. In this study, perceived value is mainly determined by customers' perceived gain and rendition. Customers will comprehensively measure their perceived gains and losses and finally judge their perceived value. A 5-point Likert scale is adopted for measurement, in which (1) represented “strongly disagree” and (5) represented “strongly agree.” Four items for perceived value (PV) are based on the version of Wang et al. [27] and adjusted and modified appropriately according to the context of online learning platform, as shown in Table 8.

#### 3.2.4. Measurement of Adjusting Variables

Online comments are a moderating variable of this study. Different from the way of information transmission in the real society under the influence of teachers, online comments achieve the transmission of information through online comments and then influence the decision-making behavior of customers. As network comments in external situation factors, 5-point Likert scale is applied in measurement, and the anchoring range ranges from “strongly disagree” (1) to “strongly agree” (5). Four items are based on the version of Zhao et al. [26] and adjusted and modified appropriately according to the context that parents of online learning platform could easily understand, as shown in Table 9.

## 4. Questionnaire Delivery and Data Collection

### 4.1. Distributing and Collecting Questionnaires

The questionnaire consisted of two main parts: basic information and the structure of the paper research. The former looks at the respondents' gender, age, education level, and economic status, while the second focuses on parents' sentiments toward online learning platform aspects.

The online survey platform (Wenjuanxing) distributed 900 questionnaires, and 792 were collected. After processing the sample data, 745 appropriate data samples for empirical analysis were found. The questionnaire recovery rate was 88 percent, while the effective rate was 94 percent. The following criteria were used to determine whether a questionnaire was invalid: too many items have been missed; all the answers are the same; there are obvious contradictory reactions before and after the questions.

RETRACTED

### 4.2. Sample Description

Sample population statistics are shown in Table 10, in which the male to female ratio is roughly 1 : 3, 191 men (25.6%) and 554 women (74.4%), which mirrors the fact that the education of children in China is mostly undertaken by mothers. The analysis shows that there is no significant difference between the families where mothers undertake the children's education and those where fathers undertake it, which does not affect the study. In order to improve the coverage rate of samples, this study deliberately selected some counties and towns schools for investigation. Most middle school students' parents have junior high school (49.5%) or junior college/bachelor's diploma (32.6%) (32.6%), aged 36–45 years old, accounting for 73.1%, and over half of the families earn less than 5,000 yuan each month. Through the analysis of the questionnaire, it is concluded that no marked difference among students' parents in rural and urban schools in their investment in their children's learning is found, and no marked difference between students' parents with higher and lower education is found. The survey also found some low-income families, whose investment in children's learning is “huge,” and there is no significant difference with high-income families. The sample was adequate for this study given the ratio of sample size to items [30].

Descriptive statistics were analyzed for the measurement items in this study.  Table 11 presents the results.  Table 11 covers the maximum, minimum, mean, and standard deviation for all items in the eight variables of perceived usefulness, platform information, perceived risk, perceived cost, online comments, teacher influence, perceived value, and parent attitude, as well as skewness coefficient and kurtosis coefficient describing data distribution state. From the skewness coefficient, it is found that the parameters are generally negative, and the data generally show a trend of left skewness. It can be seen from the kurtosis coefficient that the kurtosis coefficient is generally below 0, indicating the entire data distribution is relatively average in comparison with normal distribution and has a flat peak. Thus, it can be said that the data in this study do not conform to the standard multivariate normal distribution.

### 4.3. Data Analysis Methods

According to the research purpose, research content, research object, theoretical model, research hypothesis, and sample data, the authors adopt the following three empirical research data analysis methods.

#### 4.3.1. Descriptive Statistical Analysis

Descriptive statistical analysis aims to analyze and explain the overall characteristics of the data samples, so as to have a more accurate and detailed understanding of the overall characteristics of the samples and data, such as gender, education level, age range, and monthly income level in respondents. At the same time, this method also comprehensively describes the basic characteristics and distribution of sample data, such as the frequency number, frequency, and cumulative percentage of variables or attributes in the sample, and forms a preliminary judgment before in-depth analysis of the data. Data analysis software SPSS Statistics 22.0 was used in this study.

RETRACTED

#### 4.3.2. Reliability and Validity Analysis

Reliability and validity analysis shows the authenticity and accuracy of sample data used to measure the study variables. Reliability analysis is mainly concerned with measuring the stability of the measurement target structure, that is, if repeated measurements under similar conditions can produce reliable and stable measurement findings. Reliability is defined as the extent to which a measurement tool is free from the influence of random errors. Validity is mainly to determine whether the scale can really measure constructs [31], which mainly refers to the accuracy of measurement. High reliability means small random error, while high efficiency means small random error and systematic error. Reliability is a necessary condition for validity. If a measurement value is unreliable, it cannot be valid. However, reliability is not an adequate qualification for validity, because even if the random error is zero, there may still be systematic error. Therefore, although the measured value has good consistency and stability, it may still deviate from the true value. AMOS 24.0 and SPSS 22.0 are used for confirmatory factor analysis to calculate the standardized factor load, item reliability, component reliability, convergence validity, and discriminant validity of each variable scale to ensure that the scale measured the research construct. The specific results are detailed in the latter part of this chapter.

#### 4.3.3. Structural Equation Model

Structural equation model (SEM) has obtained wide application in management research. This method is a combination of regression analysis, factor analysis, and path analysis and other statistical analysis methods, through statistical analysis, to test and explain the causality of research variables, and a measurement model is established. And the latent variable is measured with the help of a structured way, with the help of a structural model of the theory of structural relations of latent variables to construct. The complicated relation among numerous variables and multiple measurement errors can be processed and analyzed simultaneously. In conclusion, this study uses SPSS 22.0 AMOS 24.0 software to investigate the structural equation model. When estimating the structural equation model, the structural equation model's correctness was verified by the model fit.

RETRACTED

#### 4.3.4. Mediating Effect

In this study, the direct effect, indirect effect, and total effect of the path are deeply analyzed when the mediation effect of variables is tested. Bootstrapping method is employed for exploring the mediation effect of variables. In general, the most widely used approach is the Casual Steps Approach proposed by Baron and Kenny in 1986, which requires researchers to estimate each path in a model and determine whether variables act as mediators based on statistical criteria [32]. Although this method is relatively simple and widely understood, it has been severely criticized by scholars in many aspects [33, 34]. Another mediation analysis method commonly used at present is Sobel Test [35]. A fatal flaw in Sobel test lies in its assumption for the normal sampling distribution of indirect effects, whereas AB sampling distribution is asymmetric. The Sobel Test method, while being useful, is often used as a complement to Baron and Kenny rather than a replacement. Therefore, Bootstrapping is a more reasonable research method to study the mediation effect in this paper. At present, Bootstrapping has been implemented in some SEM software, such as Mplus, AMOS, and EQS. Studies show that Bootstrapping is better than Sobel test and causal step method to predict the mediating relationship between variables [36].

### 4.4. Data Analysis and Hypothesis Testing

#### 4.4.1. Exploratory Factor Analysis

*(1) Exploratory Factor Analysis of Perceived Usefulness*. According to Table 12, the KMO value for exploratory factor analysis sample used for perceived usefulness is 0.726, greater than the minimum standard value of 0.5. The chi-square value in Bartlett's spherical test is 1796.925, with a degree of freedom of 3, and has passed the significance test, indicating good data quality and suitable for exploratory factor analysis. Through exploratory analysis, a factor structure with an eigenvalue of 2.581 > 1 was obtained. The factor loading values of item PU1, PU2, and PU3 were 0.947, 0.887, and 0.947, respectively, which exceeded the minimum standard value of 0.5, and accounted for 86.03% of the variance variation, which was greater than 50% of the minimum standard value. Therefore, the factor structure of the perceived usefulness variable can be judged to be consistent with the preset structure.

*(2) Exploratory Factor Analysis of Platform Information*. According to Table 13, the KMO value for exploratory factor analysis sample used for platform information is 0.671, above the minimum standard value of 0.5. The chi-square value of Bartlett's spherical test is 1054.302, with a degree of freedom of 3, and it has passed the significance test, indicating good data quality and suitable for exploratory factor analysis. Through exploratory analysis, a factor structure with an eigenvalue of 2.268 > 1 was obtained. The factor loading values of PI1, PI2, and PI3 were 0.782, 0.908, and 0.912, respectively, above the minimum standard value of 0.5, explaining 75.61% of the variance variation and greater than 50% of the minimum standard value. Therefore, it can be judged that the factor structure of the platform information variable is consistent with the preset structure.

*(3) Exploratory Factor Analysis of Perceived Risk*. According to Table 14, the KMO value for exploratory factor analysis sample used for perceived risk is 0.705, greater than the minimum standard value of 0.5. The chi-square value of Bartlett's spherical test is 686.901, with a degree of freedom of 3, and it has passed the significance test, indicating good data quality and suitable for exploratory factor analysis. Through exploratory analysis, a factor structure with characteristic value of 2.134 > 1 was obtained. The factor loading values of PR1, PR2, and PR3 were 0.831, 0.834, and 0.864, respectively, which exceeded the minimum standard value of 0.5, and accounted for 71.12% of the variance variation and more than 50% of the minimum standard value. Therefore, it can be judged that the factor structure of perceived risk variable is consistent with the preset structure.

*(4) Exploratory Factor Analysis of Perceived Cost*. According to Table 15, the KMO value for exploratory factor analysis sample used for perceived cost is 0.743, exceeding the minimum standard value of 0.5. The chi-square value of Bartlett's spherical test is 1012.681, with a degree of freedom of 6, and has passed the significance test, indicating good data quality and suitable for exploratory factor analysis. Through exploratory analysis, a factor structure with characteristic value of 2.537 > 1 was obtained. The factor loading values of PC1, PC2, PC3, and PC4 were 0.827, 0.768, 0.767, and 0.822, respectively, which exceeded the minimum standard value of 0.5, explaining 63.43% of the variance variation and greater than 50% of the minimum standard value. Therefore, it can be judged that the factor structure of the perceived cost variable is consistent with the preset structure.

*(5) Exploratory Factor Analysis of Teacher Influence*. According to Table 16, the KMO value for exploratory factor analysis sample used for teacher influence is 0.804, exceeding the minimum standard value of 0.5. The chi-square value of Bartlett's spherical test is 1340.387, with a degree of freedom of 6, and it has passed the significance test, indicating good data quality and suitable for exploratory factor analysis. Through exploratory analysis, a factor structure with characteristic value of 2.809 > 1 was obtained. The factor loading values of TI1, TI2, TI3, and TI4 were 0.870, 0.809, 0.834, and 0.838, respectively, which exceeded the minimum standard value of 0.5, and accounted for 70.21% of the variance variation and more than 50% of the minimum standard value. Therefore, it can be judged that the factor structure of teacher influence variable is consistent with the preset structure.

*(6) Exploratory Factor Analysis of Network Comments*. According to Table 17, the KMO value for exploratory factor analysis sample used for online reviews is 0.743, exceeding the minimum standard value of 0.5. The chi-square value of Bartlett's spherical test is 951.353, with a degree of freedom of 6, and it has passed the significance test, indicating good data quality and suitable for exploratory factor analysis. Through exploratory analysis, a factor structure with characteristic value of 2.509 > 1 was obtained. The factor loading values of OC1, OC2, OC3, and OC4 were 0.774, 0.825, 0.829, and 0.736, respectively, which exceeded the minimum standard value of 0.5, explaining 62.72% of the variance variation and greater than 50% of the minimum standard value. Therefore, it can be judged that the factor structure of the network comment variable is consistent with the preset structure.

*(7) Exploratory Factor Analysis of Perceived Value*. According to Table 18, the KMO value for exploratory factor analysis sample used for perceived value is 0.808, greater than the minimum standard value of 0.5. The chi-square value of Bartlett's spherical test is 2119.720, with a degree of freedom of 6, and it has passed the significance test, indicating good data quality and suitable for exploratory factor analysis. Through exploratory analysis, a factor structure with a characteristic value of 3.154 > 1 was obtained. The factor loading values of item PV1, PV2, PV3, and PV4 were 0.863, 0.884, 0.905, and 0.899, respectively, which exceeded the minimum standard value of 0.5, and accounted for 78.85% of the total variance variation, which was greater than 50% of the minimum standard value. Therefore, it can be judged that the factor structure of the perceived value variable is consistent with the preset structure.

*(8) Exploratory Factor Analysis of Parents' Attitude*. According to Table 19, the KMO value for exploratory factor analysis sample used for parents' attitudes is 0.756, greater than the minimum standard value of 0.5. The chi-square value of Bartlett's spherical test is 1559.966, with a degree of freedom of 3, and it has passed the significance test, indicating good data quality and suitable for exploratory factor analysis. Through exploratory analysis, a factor structure with a characteristic value of 2.559 > 1 was obtained. The factor loading values of item PA1, PA2, and PA3 were 0.922, 0.934, and 0.914, respectively, which exceeded the minimum standard value of 0.5, and accounted for 85.31% of the variance variation, which was higher than 50% of the minimum standard value. Therefore, it can be determined that the factor structure of parental attitude variable is consistent with the preset structure.

RETRACTED

#### 4.4.2. Model Testing

To examine the link between putative observed variables and putative potential variables, confirmatory factor analysis (CFA) is performed under the measurement model using AMOS24.0 and SPSS 22.0. Platform information, perceived usefulness, perceived risk, perceived cost, teacher influence, perceived value, online comments, and parent attitudes were all subjected to CFA analysis. Tables 20 and 21 summarize the findings. The standardized factor loadings of all eight dimensions are above 0.6 and signed, and the question reliability is above 0.36. The 8 dimensions' constituent reliability is more than 0.7, showing high internal consistency. The convergence validity (mean variance extraction amount) exceeding 0.5 proved the favorable convergence effect. The research results meet the criteria of factor load higher than 0.5, composition reliability higher than 0.6, and convergence validity higher than 0.5 proposed by Fornell and Larcker [37] and Hair et al. [38]. By analyzing the association between the AVE square root value and other dimensions, the discriminant validity is verified. In this study, eight variables, including independent variable, intermediary variable, moderating variable, and dependent variable, are studied for discriminant validity.  Table 21 shows the results. Except for the AVE square root value of teacher influence, which is relatively lower than the correlation coefficient with network comments, all other AVE square root values in the matrix are higher than the correlation coefficient between the AVE square root value and associated dimensions. As THE AVE method is a relatively rigorous method for determining discriminant validity, generally speaking, the results of discriminant validity are acceptable.

The constructed model is measured by two types of fitting indexes: absolute fit index and value-added fit index. *χ*^2^/ DF, GFI, AGFI, and RMSEA are all part of the absolute fitness index. The value-added fitness indexes are NFI, RFI, IFI, TLI, and CFI. It is impossible for data in SEM analysis to correspond to a multivariate normal distribution [39], while nonmultivariate normal is easy to cause *χ*^2^ inflation. Therefore, Bollen-Stine Bootstrap *p* procedure is used in this paper to compensate for the lack of multivariate normality, and the model fitting and parameter estimation must be adjusted [40, 41]. After modification, the findings are presented in in Table 22, and the absolute fitness index and value-added fitness index basically present a good situation.

RETRACTED

#### 4.4.3. Impact Path Test

As shown in Table 23 and Figure 2, perceived usefulness significantly positively affects parent attitudes (PU⟶PA: *β* = 0.687, *t* = 18.301, *P* < 0.001), supporting Hypothesis 1. Perceived usefulness positively significantly affects perceived value (PU⟶PV: *β* = 0.406, *t* = 12.132, *P* < 0.001). Hypothesis 2 is true. Platform information positively affected parent attitude (PI⟶PA: *β* = 0.106, *t* = 3.050, *P* < 0.01). Hypothesis 3 is true. Platform information significantly positively affects perceived value (PI⟶PV: *β* = 0.458, *T* = 12.689, *P* < 0.001), and hypothesis 4 is true. Hypotheses 1–4 indicate that the perceived usefulness and platform information as perceived benefits have a favorable effect on perceived value and parent attitudes. Perceived risk has a significant negative effect on perceived value (PR⟶PV: *β* = −0.153, *t* = −4.688, *P* < 0.001). Hypothesis 5 is true. Perceived risk significantly negatively affects parent attitudes (PR⟶PA: *β* = −0.088, *t* = −3.217, *P* < 0.01). Hypothesis 6 is true. Perceived cost has no significant negative influence on perceived value (PC⟶PV: *β* = −0.051, *t* = −1.630, *P*=0.103 > 0.05), and hypothesis 7 is not true. Perceived cost significantly positively affects parents' attitudes (PC⟶PA: *β* = 0.161, *t* = 5.936, *P* < 0.001), contrary to hypothesis 8, which is not valid. Hypothesis 5 assumes that the establishment of the 6 shows the negative influence perceived risk as part of the benefit of perception value perception and attitude of parents, but assumptions 7 and 8 do not explain the perceived costs as part of the perceived benefit of not negative influence perceived value and attitude of parents, and perceived cost does not significantly affect online learning platform use. Teacher influence has a significant positive impact on perceived value (TI⟶PV: *β* = 0.481, *T* = 12.397, *P* < 0.001). Hypothesis 9 is true. The influence of teachers significantly positively affects parents' attitudes (TI⟶PA: *β* = 0.279, *T* = 7.384, *P* < 0.001). Hypothesis 10 is true. Teacher influence as a third party environmental factor of online learning platform influences the connection between parents of middle school students and online learning platforms. Perceived value significantly positively affects parent attitude (PV⟶PA: *β* = 0.191, *t* = 3.811, *P* < 0.001). Hypothesis 12 is supported.

RETRACTED

*R* ^2^ is one of the main criteria used to evaluate the path of a structural model. This coefficient measures the model's predictive power and computes the variance of real and predicted values of a particular endogenous variable, which is the sum of the changes caused by all exogenous variables. Larger *R*^2^ indicates the model's stronger explanatory power. As shown in Figure 2, the *R*^2^ value of the endogenous variable of perceived value is 0.63, which is between 0.33 and 0.67, indicating that the model has a moderate degree of explanation. The *R*^2^ value of the endogenous variable of parents' attitude is 0.81 greater than 0.67, indicating that the model had a high degree of explanation.

#### 4.4.4. Mediating Effect Test

In addition to testing the proposed hypothesis, this study tests the mediation effect of variables and conducts in-depth analysis of the direct effect, indirect effect, and total effect of the path. Bootstrapping method is employed for exploring variable mediation effect. In this study, AMOS24 software is used to resample 2000 times under 95% confidence interval for Bootstrapping analysis of variables [42].

The nonstandardized direct effect, indirect effect, and total effect are analyzed under the hypothetical model.  Table 24 presents the findings. The model assumes that five independent variables, including perceived usefulness, platform information, perceived risk, perceived cost, and teacher influence, both directly affect parent attitudes and indirectly affect parent attitudes through perceived value. In the Perceived usefulness (PU) ⟶ Parent attitude (PA) path, as *Z* = 10.400 is greater than threshold 1.96, and the range of bias-corrected and Percentile excludes 0, it can be seen that the direct effect of perceived usefulness (PU) ⟶ Parent attitude (PA) path exists. In the Perceived usefulness (PU) ⟶ perceived value (PV) ⟶ Parent attitude (PA) path, ss *Z* = 2.524 is greater than threshold 1.96, and the range of bias-corrected and Percentile excludes 0; therefore, the indirect effect of perceived usefulness (PU) ⟶ perceived value (PV) ⟶ parent attitude (PA) exists. The total effect from perceived usefulness (PU) to parental attitude (PA) also exists (*Z* = 11.841 > 1.96, and the range of Bias-corrected and Percentile excludes 0). At this point, perceived value is a partial mediation between perceived usefulness (PU) and parental attitude (PA). In the Platform information (PI) ⟶ Parent attitude (PA) path, ss *Z* = 2.026 is greater than threshold 1.96, and the range of bias-corrected and Percentile excludes 0. The direct effect of platform information (PI) ⟶ parent attitude (PA) path exists. In the Platform information (PI) ⟶ perceived value (PV) ⟶ Parent attitude (PA) path, as *Z* = 2.538 > 1.96, and bias-corrected and Percentile ranges do not contain 0, it can be seen that the indirect effect of platform information (PI) ⟶ perceived value (PV) ⟶ parent attitude (PA) path exists. The total effect of platform information (PI) ⟶ parent attitude (PA) also exists (*Z* = 4.394 > 1.96, and bias-corrected and Percentile ranges do not contain 0). At this point, perceived value serves as a partial intermediary between platform information (PI) and parent attitude (PA).

RETRACTED

In the Perceived risk (PR) ⟶ Parent attitude (PA) path, as the absolute value of *Z* = -2.333 is greater than threshold 1.96, the range of bias-corrected and Percentile excludes 0. The direct effect of perceived risk (PR) ⟶ parent attitude (PA) path exists. In the Perceived risk (PR) ⟶ perceived value (PV) ⟶ Parent attitude (PA) path, as the absolute value of *Z* = −2.111 is above 1.96, the range of bias-corrected and Percentile excludes 0. Thus, the indirect effect of perceived risk (PR) ⟶ perceived value (PV) ⟶ parent attitude (PA) exists. The total effect of perceived risk (PR) ⟶ parental attitude (PA) also exists (*Z* = −3.125, the absolute value of *Z* is above 1.96, and the range of bias-corrected and Percentile excludes 0). At this point, perceived value is a partial intermediary between perceived risk (PR) and parental attitude (PA). As the hypothesis of the path of perceived cost (PC) ⟶ parent attitude (PA) has been proved to be invalid in the hypothesis testing above, the mediating effect of perceived cost (PC) ⟶ parent attitude (PA) is not analyzed.

In the Teacher influence (TI) ⟶ Parent attitude (PA) path, as *Z* = 3.607 is greater than threshold 1.96, the range of bias-corrected and Percentile excludes 0. Thus, the direct effect of teacher influence (TI) ⟶ parent attitude (PA) path exists. In the Teacher influence (TI) ⟶ perceived value (PV) ⟶ Parent attitude (PA) path, as *Z* = 2.607 > 1.96, the range of bias-corrected and Percentile excludes 0. Thus, the indirect effects of teacher influence (TI) ⟶ perceived value (PV) ⟶ parent attitude (PA) path exist. The total effect of teacher influence (TI) ⟶ parent attitude (PA) also exists (*Z* = 5.309 > 1.96, and the range of bias-corrected and Percentile excludes 0). At this point, perceived value is a partial intermediary between teacher influence (TI) and parent attitude (PA).

RETRACTED

In conclusion, perceived value can in part mediate the relation between perceived gain factors (perceived usefulness and platform information) and dependent variables (parent attitudes), while perceived value can in part mediate the relation between perceived loss (perceived risk) and dependent variables (parent attitudes). Perceived value can also in part mediate the relation between the external environmental variable (teacher's influence) and the dependent variable (parent attitude). It can be seen that perceived value as an important part of the mediation variable in the study of parent attitudes towards online learning platforms affects the connection between independent variables and dependent variables.

#### 4.4.5. Test of Regulatory Effect

In general, there is some difficulty in using potential variables when analyzing interactions through structural equations. Upon detecting the impacts of the interaction, nonlinear constraints should be firstly imposed on fixed factor coefficients and error variances. Second, whether indicators for the interaction term are normally distributed can be hardly confirmed even if every variable that makes up the interaction term is present. To address the above issues and explore the moderating relationship between online reviews on perceived value and parental attitudes, AMOS 24.0 adopts the two-step technique proposed by PING, eliminating the nonlinear constraint [43]. As seen in Figure 3 and Table 25, PXO, the interaction term between perceived value and online reviews, has a significant positive effect on parent attitudes. Hypothesis 11 is true, so it can be seen that online reviews influence the relationship between perceived value and parental attitudes in a favorable way.

Through the above SPSS analysis and AMOS verification, we obtained the results for empirical research (Figure 4).

## 5. Results and Discussion

### 5.1. The Results Show the Following

1. The two variables of perceived gain have a positive and significant effect on perceived value and parent attitude. Perceived usefulness significantly positively affects parents' attitude (PU⟶PA: *β* = 0.687, *T* = 18.301, *P* < 0.001), and perceived usefulness significantly positively affects perceived value (PU⟶PV: *β* = 0.406, *T* = 12.132, *P* < 0.001). Platform information significantly positively affects parents' attitude (PI⟶PA: *β* = 0.106, *T* = 3.050, *P* < 0.01), and platform information significantly positively affects perceived value (PI⟶PV: *β* = 0.458, *T* = 12.689, *P* < 0.001).
2. Perceived profit and loss are composed of perceived risk and perceived cost. Perceived risk significantly negatively affects perceived value (PR⟶PV: *β* = −0.153, *t* = −4.688, *P* < 0.001), and perceived risk significantly negatively affects parents' attitude (PR⟶PA: *β* = −0.088, *t* = −3.217, *P* < 0.01). However, perceived cost has no significant negative influence on perceived value (PC⟶PV: *β* = −0.051, *T* = −1.630, *P*=0.103 > 0.05), and perceived cost has a significant positive influence on parents' attitude (PC⟶PA: *β* = 0.161, *t* = 5.936, *P* < 0.001), contrary to the original hypothesis, so the result is not valid. As a part of perceived profit and loss, perceived cost does not negatively affect perceived value and parents' attitudes, indicating the insignificant effect of perceived cost on online learning platform use. Therefore, middle school students' parents are more concerned about if their children can learn useful knowledge on online learning platforms, rather than the perceived cost.
3. The influence of teachers on social factors significantly positively affects perceived value (TI⟶PV: *β* = 0.481, *T* = 12.397, *P* < 0.001), and the influence of teachers on parents' attitude (TI⟶PA: *β* = 0.279, *T* = 7.384, *P* < 0.001). Teacher influence as the third party environmental factors of online learning platform influences the relationship between middle school students' parents and online learning platforms.
4. Social variables and online comments positively moderate the relation between perceived value and parent attitudes, and the interaction terms of perceived value and online comments positively affected parent attitudes (PXO⟶PA: *t* = 6.454, *P* < 0.001). Therefore, creating positive online comments during the publicity process of the online learning platform is helpful in shaping the corporate image and enhancing the perceived value and recognition of parents.
5. As a partial intermediary, perceived value influences the relationship between perceived gain variables (perceived usefulness and platform information), perceived loss variables (perceived risk), and dependent variables (parental attitude). Perceived value also partially mediates the relationship between the external environmental variable (teacher's influence) and the dependent variable (parent's attitude). It can be seen that perceived value as an important part of the mediation variable in the study of parent attitudes towards online learning platforms affects the relation between independent variables and dependent variables. Therefore, for online learning platforms, it is extremely important for parents of middle school students to perceive the value of learning, which can help improve their attitude towards online learning platforms.

RETRACTED

## 6. Conclusion

This part mainly discusses the influencing factors of parents' attitude towards secondary school students' online learning platform. Based on the theory of perceived value, the factor model of parents' attitude of secondary school students' online learning platform is established from the subjective dimension and social factor dimension. Through the questionnaire survey of parents' attitude towards secondary school students in online learning platform, 745 valid questionnaires are analyzed by structural equation model and regression analysis. The main research findings are as follows:

1. Perceived value plays an intermediary role in this research model. Perceived usefulness, platform information, and perceived risk not only influence parents' attitude directly and positively, but also indirectly influence parents' attitude through perceived value.
2. Perceived cost does not have a direct negative influence on parents' attitude, nor does it have an indirect influence on parents' attitude through perceived value.
3. The moderating effect of online comments is established. Teachers, the influencing factor of external situation, influence parents' attitude towards online learning platform through perceived value, both directly and indirectly.

## Figures and Tables

**Figure 1:** Model and hypothesis.

**Figure 2:** Hypothesis test results. Note: (1) ^*∗∗∗*^means *P* < 0.001; ^*∗∗*^means *P* < 0.01; ^*∗*^means *P* < 0.05.

**Figure 3:** Moderating model of online reviews.

**Figure 4:** Final test results. Note: (1) ^*∗∗∗*^means *P* < 0.001; ^*∗∗*^means *P* < 0.01; ^*∗*^means *P* < 0.05.

**Table 1:** Research hypotheses.

SN	Hypothesis content
H1	Parents' perceived usefulness of e-learning platforms positively affects parents' attitudes.
H2	Parents' perceived usefulness of e-learning platforms positively affects parents' perceived value.
H3	The information of online learning platform positively affects the attitudes of parents of middle school students.
H4	The information of online learning positively affects the perceived value of parents of middle school students.
H5	Perceived risk negatively affects parents' perceived value for online learning platforms.
H6	Perceived risk negatively affects the attitudes of parents of middle school students for online learning platforms.
H7	Perceived cost negatively affects parents' perceived value for online learning platforms.
H8	Perceived cost negatively affects parents' attitudes towards online learning platforms.
H9	The perceived value of online learning platforms from parents of middle school students was positively affected by teacher influence.
H10	The attitudes towards online learning platform from parents of middle school students were positively affected by teacher influence.
H11	Online comments positively moderate perceived value and parents' attitudes on online learning platforms.
H12	Perceived value positively affects the attitudes of parents of middle school students towards online learning platforms.

RETRACTED

**Table 2:** Measurement scale of perceived usefulness.

Latent variables	Item code	Questionnaire content design	Source
Perceived usefulness	PU1	Online learning platforms currently in use can improve children's learning results.	Davis [24]
	PU2	Online learning platforms are being used to meet the needs of children.	
	PU3	Online learning platforms are being used to solve children's learning puzzles.	

**Table 3:** Measurement scale of platform information.

Latent variables	Item code	Questionnaire content design	Source
Platform information	PI1	The online learning platform is rich in resources and can satisfy children's learning needs.	Li [25]
	PI2	The video quality of online learning platform is high and can satisfy children's learning needs.	
	PI3	The online learning platform is rich in information about courses, which is helpful for children to learn.	

**Table 4:** Measurement scale of perceived risk.

Latent variables	Item code	Questionnaire content design	Source
Perceived risk	PR1	Online learning platform course content does not match the description, and the quality of the course is not up to standard.	Zhao et al. [26]
	PR2	Children use online learning platform to learn courses, and the learning effect is not obvious.	
	PR3	Online learning platform related content offline services are not guaranteed.	

**Table 5:** Measurement scale of perceived cost.

Latent variables	Item code	Questionnaire content design	Source
Perceived cost	PC1	Online learning platforms require additional purchase of expensive learning equipment.	Wang et al. [27]
	PC2	Online learning platforms take children more time to get used to and be familiar with.	
	PC3	Online learning platforms have other hidden and additional fees.	
	PC4	Online learning platforms require parents to spend a lot of time and energy monitoring their children's learning process.	

**Table 6:** Measurement scale of teacher influence.

Latent variables	Item code	Questionnaire content design	Source
Teacher influence	TI1	The course content of the online learning platform currently in use is recognized by the school teachers.	Ashwin et al. [28]
	TI2	Teachers in the school recognize the curriculum design and teaching methods of the online learning platform.	
	TI3	School teachers support online learning after school.	
	TI4	School teachers see online learning as a useful complement to classroom learning.	

RETRACTED

**Table 7:** Measurement scale of parents' use intention.

Latent variables	Item code	Questionnaire content design	Source
Parent attitude	PA1	I am willing to spend more money to choose and use effective online learning platforms.	Raghu et al. [29]
	PA2	I want to take more time to help children choose and use online learning platforms.	
	PA3	I will create a good learning environment and support children to use the online learning platform.	

**Table 8:** Measurement scale of perceived value.

Latent variables	Item code	Questionnaire content design	Source
Perceived value	PV1	Children learn better when they use online learning platforms.	Wang et al. [27]
	PV2	Online learning platforms provide targeted services for children.	
	PV3	Using online learning platforms, children can learn key knowledge more efficiently.	
	PV4	Online learning platform helps children to quickly find the right learning content.	

**Table 9:** Measurement scale of online comments.

Latent variables	Item code	Questionnaire content design	Source
Online comment	OC1	When choosing an online learning platform, I refer to other people's comments.	Zhao et al. [26]
	OC2	I prefer to let kids use online learning platforms with good reviews on content.	
	OC3	I prefer to use an online learning platform with a famous teacher.	
	OC4	Negative comments will affect my choice and use of online learning platforms.	

**Table 10:** Demographic data.

Population profile	Category	Frequency number	Frequency	Cumulative percentage (%)
Gender	Male	191	25.6	25.6
	Female	554	74.4	100.0

Education level	Master or above	14	1.9	1.9
	Junior college/undergraduate	243	32.6	34.5
	Senior middle school	119	16.0	50.5
	Junior middle school	369	49.5	100.0

Age range	30–35	52	7.0	7.0
	36–40	238	31.9	38.9
	41–45	255	34.2	73.2
	46–50	135	18.1	91.3
	Others	65	8.7	100.0

Monthly income level	8000 above	63	8.5	8.5
	6500–8000	41	5.5	14.0
	5000–6500	88	11.8	25.8
	3500–5000	208	27.9	53.7
	2000–3500	345	46.3	100.0

**Table 11:** Descriptive statistics of items.

	*N*	Min	Max	Mean	SD	Skewness		Kurtosis	
	Statistics	Statistics	Statistics	Statistics	Statistics	Statistics	SE	Statistics	SE
PU1	745	1.000	5.000	3.790	1.158	−0.683	0.090	−0.198	0.179
PU2	745	1.000	5.000	3.880	1.147	−0.785	0.090	−0.076	0.179
PU3	745	1.000	5.000	3.740	1.154	−0.613	0.090	−0.250	0.179
PI1	745	1.000	5.000	3.690	1.121	−0.489	0.090	−0.309	0.179
PI2	745	1.000	5.000	3.730	1.145	−0.488	0.090	−0.511	0.179
PI3	745	1.000	5.000	3.850	1.097	−0.625	0.090	−0.247	0.179
PR1	745	1.000	5.000	2.650	1.384	0.294	0.090	−1.114	0.179
PR2	745	1.000	5.000	2.910	1.304	0.100	0.090	−0.983	0.179
PR3	745	1.000	5.000	2.980	1.426	−0.004	0.090	−1.267	0.179
PC1	745	1.000	5.000	3.830	1.206	−0.782	0.090	−0.261	0.179
PC2	745	1.000	5.000	4.100	1.128	−1.090	0.090	0.366	0.179
PC3	745	1.000	5.000	3.590	1.276	−0.532	0.090	−0.671	0.179
PC4	745	1.000	5.000	3.820	1.159	−0.656	0.090	−0.360	0.179
TI1	745	1.000	5.000	3.570	1.185	−0.438	0.090	−0.458	0.179
TI2	745	1.000	5.000	3.750	1.151	−0.602	0.090	−0.363	0.179
TI3	745	1.000	5.000	3.380	1.217	−0.252	0.090	−0.645	0.179
TI4	745	1.000	5.000	3.780	1.161	−0.673	0.090	−0.243	0.179
PV1	745	1.000	5.000	3.370	1.081	−0.117	0.090	−0.245	0.179
PV2	745	1.000	5.000	3.520	1.111	−0.262	0.090	−0.428	0.179
PV3	745	1.000	5.000	3.570	1.121	−0.296	0.090	−0.485	0.179
PV4	745	1.000	5.000	3.590	1.114	−0.327	0.090	−0.424	0.179
OC1	745	1.000	5.000	3.580	1.231	−0.458	0.090	−0.628	0.179
OC2	745	1.000	5.000	3.470	1.234	−0.362	0.090	−0.671	0.179
OC3	745	1.000	5.000	3.490	1.212	−0.397	0.090	−0.541	0.179
OC4	745	1.000	5.000	3.740	1.158	−0.613	0.090	−0.267	0.179
PA1	745	1.000	5.000	3.800	1.125	−0.654	0.090	−0.194	0.179
PA2	745	1.000	5.000	3.880	1.116	−0.717	0.090	−0.143	0.179
PA3	745	1.000	5.000	3.830	1.138	−0.730	0.090	−0.092	0.179

RETRACTED

**Table 12:** Results of exploratory factor analysis of perceived usefulness.

Item code	Perceived usefulness
PU1	0.947
PU2	0.887
PU3	0.947
Eigenvalue	2.581
Cumulative variation interpretation	86.03%
KMO value = 0.726	
Bartlett's spherical test chi-square value = 1796.925	
DOF = 3	
(Sig.) *p*=0.000	

**Table 13:** Results of exploratory factor analysis of platform information.

Item code	Platform information
PI1	0.782
PI2	0.908
PI3	0.912
Eigenvalue	2.268
Cumulative variation interpretation	75.61%
KMO value = 0.671	
Bartlett's spherical test chi-square value = 1054.302	
DOF = 3	
(Sig.) *p*=0.000	

**Table 14:** Results of exploratory factor analysis of perceived risk.

Item code	Perceived risk
PR1	0.831
PR2	0.834
PR3	0.864
Eigenvalue	2.134 (%)
Cumulative variation interpretation	71.12
KMO value = 0.705	
Bartlett's spherical test chi-square value = 686.901	
DOF = 3	
(Sig.) *p*=0.000	

**Table 15:** Results of exploratory factor analysis of perceived cost.

Item code	Perceived cost
PC1	0.827
PC2	0.768
PC3	0.767
PC4	0.822
Eigenvalue	2.537 (%)
Cumulative variation interpretation	63.43
KMO value = 0.743	
Bartlett's spherical test chi-square value = 1012.681	
DOF = 6	
(Sig.) *p*=0.000	

**Table 16:** Results of exploratory factor analysis of teacher influence.

Item code	Teacher influence
TI1	0.870
TI2	0.809
TI3	0.834
TI4	0.838
Eigenvalue	2.809
Cumulative variation interpretation	70.21%
KMO value = 0.804	
Bartlett's spherical test chi-square value = 1340.387	
DOF = 6	
(Sig.) *p*=0.000	

**Table 17:** Results of exploratory factor analysis of online comments.

Item code	Online comment
OC1	0.774
OC2	0.825
OC3	0.829
OC4	0.736
Eigenvalue	2.509
Cumulative variation interpretation	62.72%
KMO value = 0.743	
Bartlett's spherical test chi-square value = 951.353	
DOF = 6	
(Sig.) *p*=0.000	

RETRACTED

**Table 18:** Results of exploratory factor analysis of perceived value.

Item code	Perceived value
PV1	0.863
PV2	0.884
PV3	0.905
PV4	0.899
Eigenvalue	3.154
Cumulative variation interpretation	78.85%
KMO value = 0.808	
Bartlett's spherical test chi-square value = 2119.720	
DOF = 6	
(Sig.) *p*=0.000	

**Table 19:** Results of exploratory factor analysis of parents' use intention.

Item code	Parent attitude
PA1	0.922
PA2	0.934
PA3	0.914
Eigenvalue	2.559
Cumulative variation interpretation	85.31%
KMO Value = 0.756	
Bartlett's spherical test chi-square Value = 1559.966	
DOF = 3	
(Sig.) *p*=0.000	

**Table 20:** Confirmatory factor analysis results.

Dimensionality	Title	Parameter significance estimation				Standardized factor load	Title reliability	Composite reliability
		Unstd.	S.E.	*t*-value	*p*	Std.	SMC	CR
PU	PU1	1.000				0.942	0.887	0.921
	PU2	0.826	0.028	29.718	^*∗∗∗*^	0.785	0.616	
	PU3	0.998	0.023	42.638	^*∗∗∗*^	0.943	0.889	

PI	PI1	1.000				0.610	0.372	0.849
	PI2	1.484	0.085	17.559	^*∗∗∗*^	0.887	0.787	
	PI3	1.446	0.083	17.456	^*∗∗∗*^	0.902	0.814	

PR	PR1	1.000				0.720	0.518	0.798
	PR2	0.951	0.058	16.426	^*∗∗∗*^	0.726	0.527	
	PR3	1.164	0.071	16.507	^*∗∗∗*^	0.814	0.663	

PC	PC1	1.000				0.766	0.587	0.809
	PC2	0.833	0.050	16.501	^*∗∗∗*^	0.682	0.465	
	PC3	0.927	0.057	16.264	^*∗∗∗*^	0.670	0.449	
	PC4	0.939	0.053	17.677	^*∗∗∗*^	0.748	0.560	

TI	TI1	1.000				0.835	0.697	0.859
	TI2	0.854	0.041	20.813	^*∗∗∗*^	0.734	0.539	
	TI3	0.945	0.043	21.914	^*∗∗∗*^	0.769	0.591	
	TI4	0.901	0.041	21.909	^*∗∗∗*^	0.768	0.590	

PV	PV1	1.000				0.775	0.601	0.910
	PV2	1.072	0.046	23.533	^*∗∗∗*^	0.808	0.653	
	PV3	1.208	0.045	26.785	^*∗∗∗*^	0.902	0.814	
	PV4	1.189	0.045	26.522	^*∗∗∗*^	0.893	0.797	

PA	PA1	1.000				0.879	0.773	0.914
	PA2	1.031	0.031	33.263	^*∗∗∗*^	0.913	0.834	
	PA3	0.987	0.032	30.765	^*∗∗∗*^	0.857	0.734	

OC	OC1	1.000				0.663	0.440	0.803
	OC2	1.185	0.072	16.395	^*∗∗∗*^	0.783	0.613	
	OC3	1.159	0.071	16.372	^*∗∗∗*^	0.780	0.608	
	OC4	0.862	0.063	13.745	^*∗∗∗*^	0.607	0.368	

Note: (1) PU = perceived usefulness; PI = platform information; PR = perceived risk; PC = perceived cost; TI = teacher influence; PV = perceived value; PA = parent attitude; OC = online comment; Unstd. = nonstandardized factor load; S.E. = standard error; *t*-value = *t* value; NA = not available (regression coefficient fixed at 1.0); Std. = standardized factor load; SMC = topic reliability; CR = constituent reliability. (2) ^*∗∗∗*^means *P* < 0.001; *N* = 745.

**Table 21:** Validity evaluation of discriminant validity.

Dimension	Convergent validity	Discriminant validity							
	AVE	PU	PI	PR	PC	TI	OC	PV	PA
PU	0.860	**0.927**							
PI	0.756	0.694	**0.869**						
PR	0.711	−0.311	−0.289	**0.843**					
PC	0.635	0.144	0.143	0.140	**0.797**				
TI	0.702	0.722	0.708	−0.321	0.210	**0.838**			
OC	0.627	0.750	0.683	−0.319	0.271	0.843	**0.792**		
PV	0.788	0.722	0.787	−0.376	0.091	0.738	0.720	**0.888**	
PA	0.852	0.838	0.725	−0.351	0.227	0.768	0.761	0.767	**0.923**

Note: (1) PU = perceived usefulness; PI = platform information; PR = perceived risk; PC = perceived cost; TI = teacher influence; OC = online comments; PV = perceived value; PA = parental attitude; AVE = convergence validity. (2) The diagonal elements in the matrix are AVE square root values, and the nondiagonal elements represent the correlation of related dimensions.

RETRACTED

**Table 22:** Modified model fitting index.

Amount of inspection	Absolute fitness index				Value added fit index				
	*χ* ^2^/df	GFI	AGFI	RMSEA	NFI	RFI	IFI	TLI	CFI
Good standard	<3	>0.9	>0.9	<0.08	>0.9	>0.9	>0.9	>0.9	>0.9
Model	1.44	0.97	0.97	0.02	0.97	0.97	0.99	0.99	0.99

Note: this is the fitting degree of bootstrap model for 2000 times.

**Table 23:** Hypothesis test.

Hypothesis	Standardized path coefficient	Nonstandardized path coefficient	S.E.	*t*-value	*P*	Result
Hypothesis 1: PU⟶PA	0.687	0.468	0.026	18.301	^*∗∗∗*^	True
Hypothesis 2: PU⟶PV	0.406	0.239	0.020	12.132	^*∗∗∗*^	True
Hypothesis 3: PI⟶PA	0.106	0.079	0.026	3.050	^*∗∗*^	True
Hypothesis 4: PI⟶PV	0.458	0.297	0.023	12.689	^*∗∗∗*^	True
Hypothesis 5: PR⟶PV	−0.153	−0.084	0.018	−4.688	^*∗∗∗*^	True
Hypothesis 6: PR⟶PA	−0.088	−0.056	0.018	−3.217	^*∗∗*^	True
Hypothesis 7: PC⟶PV	−0.051	−0.038	0.024	−1.630	0.103	False
Hypothesis 8: PC⟶PA	0.161	0.139	0.023	5.936	^*∗∗∗*^	False
Hypothesis 9: TI⟶PV	0.481	0.327	0.026	12.397	^*∗∗∗*^	True
Hypothesis 10: TI⟶PA	0.279	0.220	0.030	7.384	^*∗∗∗*^	True
Hypothesis 12: PV⟶PA	0.191	0.221	0.058	3.811	^*∗∗∗*^	True

Note: (1) PU = perceived usefulness; PI = platform information; PR = perceived risk; PC = perceived cost; TI = teacher influence; PV = perceived value; PA = parent attitude. (2) ^*∗∗∗*^means *P* < 0.001; ^*∗∗*^means *P* < 0.01; ^*∗*^means *P* < 0.05.

**Table 24:** The mediating effect tests.

Variable	Point estimate	Product of coefficients		Bias-corrected		Percentile	
		S.E.	Z	Lower	Upper	Lower	Upper
PU->PV-->PA	0.053	0.021	2.524	0.017	0.104	0.013	0.097
PU-->PA	0.468	0.045	10.400	0.380	0.563	0.384	0.567
TOTAL EFFECT PU->PV-->PA	0.521	0.044	11.841	0.430	0.606	0.433	0.608
PI->PV-->PA	0.066	0.026	2.538	0.020	0.124	0.016	0.117
PI-->PA	0.079	0.039	2.026	0.003	0.160	0.002	0.159
TOTAL EFFECT PI->PV-->PA	0.145	0.033	4.394	0.083	0.218	0.078	0.210
PR->PV-->PA	−0.019	0.009	−2.111	−0.043	−0.005	−0.040	−0.003
PR-->PA	−0.056	0.024	−2.333	−0.104	−0.012	−0.101	−0.009
TOTAL EFFECT PR->PV-->PA	−0.075	0.024	−3.125	−0.127	−0.029	−0.122	−0.024
TI->PV-->PA	0.073	0.028	2.607	0.024	0.134	0.018	0.126
TI-->PA	0.220	0.061	3.607	0.115	0.349	0.119	0.352
TOTAL EFFECT TI->PV-->PA	0.292	0.055	5.309	0.196	0.406	0.197	0.409

Note: (1) PU = perceived usefulness; PI = platform information; PR = perceived risk; PC = perceived cost; TI = teacher influence; PV = perceived value; PA = parent attitude. (2) Unstandardized estimating of 2000 bootstrap sample.

RETRACTED

**Table 25:** Moderating effect of online reviews.

Path	Std.	S.E.	*t*-value	*P*
PV⟶PA	0.266	0.061	4.339	^*∗∗∗*^
OC⟶PA	0.611	0.064	9.508	^*∗∗∗*^
PXO⟶PA	0.039	0.006	6.454	^*∗∗∗*^

Note: (1) Std. = Standardized factor load; S.E. = standard error; *T* - value = *t* value. (2) ^*∗∗∗*^means *P* < 0.001; ^*∗∗*^means *P* < 0.01; ^*∗*^means *P* < 0.05.

## Data Availability

The experimental data used to support the findings of this study are available from the corresponding author upon request.
